# Shoutai Wan Improves Embryo Survival by Regulating Aerobic Glycolysis of Trophoblast Cells in a Mouse Model of Recurrent Spontaneous Abortion

**DOI:** 10.1155/2022/8251503

**Published:** 2022-09-28

**Authors:** Xiao Liang, Siling Tang, Dandan Li, Yajing Song, Ming He, Yancang Duan, Huilan Du

**Affiliations:** ^1^College of Integrated Traditional Chinese and Western Medicine, Hebei University of Chinese Medicine, Shijiazhuang 050091, Hebei, China; ^2^Collaborative Innovation Center of Integrated Chinese and Western Medicine on Reproductive Disease, Shijiazhuang 050091, Hebei, China; ^3^Hebei Key Laboratory of Integrative Medicine on Liver-kidney Patterns, Shijiazhuang 050091, Hebei, China

## Abstract

**Background:**

During embryo implantation, the blastocyst exhibits a high capacity for aerobic glycolysis, which results in a unique microenvironment of high lactate/low pH at the maternal-fetal interface. Shoutai Wan (STW) is an effective Chinese herbal formula widely used in the clinical treatment of recurrent spontaneous abortion (RSA). However, the specific molecular mechanism by which STW prevents abortion is yet to be elucidated.

**Methods:**

Female CBA/J mice were allocated into six groups randomly and then mated with BALB/c mice as the control group, DBA/2 mice as the RSA model, CBA/J×DBA/2 mice treated with dydrogesterone as the DQYT group, or CBA/J×DBA/2 mice treated with low, medium, and high-dose STW as the STW-L, STW-M, and STW-H groups, respectively. Drug administration started 14 days before mating and ended on the 14^th^ day of pregnancy. The embryo loss rate of each group was calculated on day 14 of gestation, and the pregnancy outcomes of the mice in each group were observed. The mouse serum was collected to determine the levels of progesterone (P) and chorionic gonadotropin (CG). The activities of HK2, PKM2, and LDHA, the key glycolytic enzymes in each group, were detected. The expressions of lactate, ATP, HK2, PKM2, LDHA, MCT4, GLUT1, and GPR81 as well as the morphology of trophoblast cells were examined.

**Results:**

The embryo loss rate and adverse pregnancy outcomes were significantly increased (*P* < 0.05) in the RSA model group. After dydrogesterone or different doses of STW treatment, the embryo loss rate and adverse pregnancy outcomes were rescued to varying degrees (*P* < 0.05). Interestingly, there was no significant difference among the groups in terms of serum P and CG (*P* < 0.05). Moreover, the activities of key glycolytic enzymes, lactate, ATP, HK2, PKM2, LDHA, MCT4, GLUT1, GPR81 protein or mRNA expression, and morphological abnormalities of trophoblast cells improved significantly in the RSA mice after dydrogesterone or different doses of STW treatment (*P* < 0.05).

**Conclusion:**

STW can promote aerobic glycolysis in trophoblast cells of RSA mouse embryos, thereby improving the microenvironment of the maternal-fetal interface and enhancing embryo implantation.

## 1. Introduction

Recurrent spontaneous abortion (RSA) is a common pregnancy complication that threatens women's physical and mental health. The recurrence risk increases with the frequency of miscarriages, and a history of spontaneous abortion is an independent risk factor for subsequent pregnancy failure. The miscarriage rates of repregnancy after one, two, and three spontaneous abortions have been reported to be 13%, 37%, and 84%, respectively [1]. The prevention and treatment of RSA have become the focus of research in the global reproductive field and have attracted wide attention from experts in various countries.

RSA belongs to the category of habitual abortion in Chinese medicine. The etiology and pathogenesis of habitual abortion are the deficiency of kidney “qi” in the human body and the deficiency of the thoroughfare channel and blood chambers; hence, the fetus cannot be nourished, which leads to embryo loss. Zhang Xichun, a famous doctor in the Qing Dynasty, believed that “the thoroughfare channel and blood chambers are the places where women conceive” and proposed that “the fertility of both men and women depends on the strength of the kidney; when kidney essence is sufficient and kidney qi is strong, the fetus is nourished.” According to the principles of reinforcing the kidney, replenishing essence, and nourishing blood, he formulated “Shoutai Wan (STW)” to treat habitual abortion. The formula consists of four herbs: *Semen Cuscutae* tonifies the kidney and replenishes essence; *Herba Taxilli* and *Radix Dipsaci* tonify the kidney and exert antiabortion effects; *Colla corii asini* nourishes the Yin and blood so that blood is plentiful in the thoroughfare-conception meridian. Many famous doctors practicing Chinese medicine have treated RSA and threatened abortion with variants of STW and achieved good clinical efficacy [2]. In recent years, research on the mechanism of STW by scholars of Chinese medicine has been deepening [3], but the specific molecular mechanism by which STW prevents miscarriage needs further exploration.

The etiology of RSA is extremely complex and diverse. Relatively definite pathogenic factors mainly include chromosomes, endocrine, infection, anatomical abnormalities of internal reproductive organs, and immunity [4]. However, the etiology remains unclear in more than 40% of clinical patients [3]. Important causes of pregnancy loss are impaired trophoblast function (migration and invasion) and embryo implantation failure [5, 6]. During early embryonic development, rapid cell proliferation and blastocoel cavity formation are dependent on significant energy and oxygen consumption. High levels of aerobic glycolysis (Warburg effect) in mammalian blastocysts, which lead to the accumulation of lactate in the extracellular microenvironment during embryo implantation, have become a well-established metabolic signature of the blastocyst [7]. The blastocyst produces high levels of lactate, and the maternal-fetal interface is relatively hypoxic during implantation. A high lactate/low pH microenvironment is thus formed around the embryo, which promotes trophoblast migration, invasion, and other blastocyst implantation processes [8]. Therefore, this study aimed to deeply investigate the molecular mechanism of STW that enhances embryo implantation by promoting aerobic glycolysis in the trophoblast cells from the perspective of the unique microenvironment of the maternal-fetal interface caused by aerobic glycolysis.

## 2. Materials and Methods

### 2.1. Medicine Preparation

The compound medicine of STW is composed of the following: *Semen Cuscutae*, *Herba Taxilli*, *Radix Dipsaci*, and *Colla corii asini* in a mass ratio of 2 : 1:1 : 1. These herbal ingredients were purchased from Shijiazhuang Lerentang Pharmaceutical Co., Ltd (China). Three different crude doses of STW were prepared 0.375, 0.75, and 1.5 g/mL, designated as STW-L (low dose), STW-M (moderate dose), and STW-H (high dose), respectively. Dydrogesterone tablets (Abbott Trading Limited, China) were milled into powder form and dissolved in 6 mL of distilled water for every 13 mg of powder to obtain the dydrogesterone solution for analysis.

### 2.2. RSA Mouse Model Establishment and Drug Treatment

Eight-week-old female CBA/J mice (*n* = 120, weight: 20–25 g), 10-week-old DBA/2 male mice (*n* = 25, weight: 35–40 g), and 10-week-old male BALB/*c* mice (*n* = 10, weight: 35–40 g) were used in this study. The mice were purchased from Liaoning Changsheng Biotechnology Co., Ltd. (certificate no. SCXK (Liao) 2017–0011). This study was approved by the Ethics Committee of the Institute of the Hebei University of Chinese Medicine (Project No: DWLL2021089, China) and conducted in accordance with the Guide for the Care and Use of Laboratory Animals (National Academy of Sciences, copyright 2010).

After a week of acclimatization, female mice with a regular estrous cycle were randomly assigned to 6 groups of 20 each as follows: control, model, dydrogesterone (DQYT), STW-L, STW-M group, and STW-H. The normal pregnancy model was established in the control group, and the RSA model was established in the other 5 groups. Female CBA/J mice and male BALB/c mice were mated in a 2 : 1 cage to create a normal pregnancy model (control group); female CBA/J mice were mated with male DBA/2 mice to create an RSA group [9]. The vaginal smear revealed a large number of sperm and combined with the observation of the vaginal opening and vaginal suppository on the first day of pregnancy. The dosage of STW-L, STW-M, and STW-H groups was 1, 2, and 4 times the clinical equivalent dose (0.83, 1.66, and 3.32 g kg^−1^ d^−1^, respectively), the dosage of the dydrogesterone group was the clinical equivalent dose (0.33 g·kg^−1^ d^−1^), and the control and model groups were provided the same volume of distilled water. Chinese medicine emphasizes the idea of “treating disease before it arises”, and the treatment of RSA focuses on “compensating weakness in advance” before the pregnancy, especially the kidneys and spleen, and protecting the fetus as soon as possible after the pregnancy occurs. Therefore, the medicine was administered continuously from 14 days before gestation to 6 and 14 days after gestation in the female mice in this study.

Eight pregnant mice were anesthetized on the 6^th^ day of pregnancy, and blood was collected from the orbit. The uterus was dissected to observe the number of embryos, and embryo tissues were collected. A part of the fetus with uterus tissues was fixed in a 4% paraformaldehyde solution, while the other tissues were stored in liquid nitrogen at −80°C. Six pregnant rats were anesthetized on the 14^th^ day of pregnancy and then injected with 0.4% trypan blue stain (Solarbio Life Sciences, China) for 30 min. Trypan blue staining revealed that the implantation site was purple-blue, and the embryos had color spots, but those not normally developed were stillborn. The total number of pregnancies was determined, and the rate of embryo loss (%) was calculated as follows: the number of stillbirths/the number of implantation staining × 100%. After the six pregnant rats gave birth naturally, we counted the litter size and the stillbirth number of each pregnant rat. Next, every 3 days, at 08:00 AM, each young rat was weighed and its length was measured until the young rats were weaned (age 21 days). During the operation, we ensured that the equipment was disinfected, and each young rat was disinfected after the measurement was completed.

### 2.3. Enzyme-Linked Immunosorbent Assay (ELISA)

Blood (1.5 mL) was collected from the retroorbital venous plexus of pregnant rats on the 6^th^ day of pregnancy, centrifuged at 4°C for 10 min at 3000 rpm, and 0.5–0.7 mL of the supernatant was taken in a test tube and stored at −80°C. The content of progesterone (P) (Elabscience, China) and chorionic gonadotropin (CG) (Shanghai Kexing Biotechnology Co., Ltd., China) in the serum was determined by using an enzyme-linked immunosorbent assay kit. The serum levels of P and CG were determined using ELISA kits according to the manufacturer's instructions.

### 2.4. Colorimetric Assay

According to the ratio of weight (g): volume (mL) = 1 : 9, adding 9 times the volume of normal saline, the sample was mechanically homogenized in an ice water bath to prepare 10% homogenate, centrifuged for 10 min at 2500 rpm, and the supernatant was collected for subsequent determination. The levels of lactate (Nanjing Jiancheng Bioengineering Institute, China), adenosine triphosphate (ATP) (Nanjing Jiancheng Bioengineering Institute, China), the activities of hexokinase (HK) (Nanjing Jiancheng Bioengineering Institute, China), pyruvate kinase (PK) (Nanjing Jiancheng Bioengineering Institute, China), and lactate dehydrogenase (LDH) (Beijing Prily Gene Technology Co., Ltd., China) in the mouse embryos were determined by a colorimetric assay according to the corresponding kit instructions.

### 2.5. HE Staining

The fetus with the mice uterus in each group were fixed with 10% formaldehyde fixative, embedded in paraffin for 24 h, and sectioned and stained with hematoxylin and eosin, and comparative observation for morphological changes of trophoblasts by optical microscopy.

### 2.6. Immunohistochemistry

Immunofluorescence double staining was performed to detect the expression of hexokinase 2 (HK2), pyruvate kinase M2 (PKM2), lactate dehydrogenase A (LDHA), monocarboxylate transporter 4 (MCT4), glucose transporter 1 (GLUT1), and G protein-coupled receptor 81 (GPR81) protein in embryonic trophoblast cells. Human trophoblast surface glycoprotein antigen 2 (TRPO2) is a specific marker of trophoblasts [10]; therefore, the target antibody was mixed with the TROP2 antibody for immunofluorescence double staining. The isolated fetus with the uterus was fixed with 4% paraformaldehyde and embedded in paraffin. The tissue paraffin sections were routinely dewaxed until hydration and then microwaved with 0.01 M sodium citrate for antigen retrieval. After incubation with 10% goat serum for 30 min to block nonspecific antigen binding, the tissue sections were incubated with anti-HK2 antibody (Abcam, USA, 1 : 400), anti-PKM2 antibody (Proteintech, China, 1 : 400), anti-LDHA antibody (Abcam, 1 : 200), anti-GLUT1 antibody (Abcam, 1 : 200), anti-MCT4 antibody (Proteintech, 1 : 100), and anti-GPR81 antibody (Novus, USA, 1 : 200) mixed with the TROP2 antibody (bio-techne, USA, 1 : 60) overnight at 4°C, followed by incubation with fluorescently labeled secondary antibodies (Proteintech, 1 : 100) in a humid chamber at 37°C for 1 h in the dark. After washing, the sections were counterstained with 4′,6-diamidino-2-phenylindole (DAPI) before observation under a fluorescence microscope (Thermo Fisher Scientific, USA). Finally, the average optical density was calculated using ImageJ, and statistical analysis was performed.

### 2.7. Quantitative Real-Time Polymerase Chain Reaction (qRT-PCR)

Total RNA Kit II (Omega Bio-Tek, USA) was used to extract the total RNA from the fetus. The purity and concentration of RNA were determined using the Nanodrop 2000C spectrophotometer (Thermo Fisher Scientific, USA). Using RNA as the template, cDNA was synthesized by reverse transcription using a reverse transcription kit (Monad, China) according to the manufacturer's instructions. Then, the SYBR Green qRT-PCR kit (Monad) was used for quantitative real-time fluorescence PCR on the Applied Biosystems 7500 Fast Real-Time PCR system (Thermo Fisher Scientific). The specific primer sequences used were as follows: *β*-actin: F: 5́́ʹ-GTGCTATGTTGCTCTAGACTTCG-3́ʹ, R: 3 ʹ -ATGCCACAGGATTCCATACC-5ʹ (117 bp); GLUT1 : F: 5ʹ-GCTTGGATCTCAGAGTCTCACGATG-3ʹ, R: 3ʹ- ATAGGGCGACGCTTGTTGAAGTATC-5ʹ (112 bp); MCT4 : F: 5ʹ-CTGGCGGTAACAGGTGAAAG-3ʹ, R: 3ʹ-CGTAGGAGAAACCCGTGATGA-5ʹ (143 bp); GPR81: 5ʹ- GGGTGGCACGATGTCATGTTCC-3ʹ, R: 3ʹ -ACCTCCTCATCCGAGCCTGTCTG-5ʹ (129 bp). All primers were designed and synthesized by Sangon Biotech (Shanghai, China) Co., Ltd. The samples to be tested were repeated in three adjacent wells to reduce operating errors, and the experiment was repeated thrice. The 2^−△△ct^ method was applied to calculate the relative quantitative value (RQ value) of the target gene expression, and the RQ value was used for statistical analysis.

### 2.8. Statistical analysis

Statistical analysis was performed using IBM SPSS 23.0. For measurement of the data, the mean ± standard deviation (SD) was employed for normally distributed measurement data, while single-factor analysis of variance (one-way ANOVA) was used to compare the mean. If the data were normally distributed, the Bonferroni test was used for data with equal variance, while Dunnett's T3 test was used to process data with unequal variance. Otherwise, the Kruskal–Wallis rank-sum test was used for non-normally distributed measurement data. The counting data were described as percentages, and the χ2 test was used. *P* < 0.05 was considered to indicate statistical significance.

## 3. Results

### 3.1. STW Improves Pregnancy Outcomes in RSA Mice

Mice in each group were sacrificed on the 14^th^ day of gestation and then dissected, and after which, the shape of the pregnant uterus was observed. In the control group, the pregnant uterus was full in shape, resembling a string of beads, with good embryo development, and the number of embryos was generally 7–9. In the model group, the aborted uterus resembled a “bamboo-like” change. After trypan blue staining, the lost embryos in the uterine cavity only demonstrated purple-blue implantation points or dark-brown blood stasis. There were 3–4 lost embryos; the absorbed embryos were smaller than the normal embryos, and their development was asynchronous. In the DQYT, STW-M, and STW-H groups, embryonic development was acceptable, and the number of normal embryos was generally about 8, of which 1–2 embryos were lost. In the STW-L group, the embryos were poorly developed, and the number of lost embryos was generally 2–3 (Figure 1). The embryo loss rate increased in the model group relative to that in the control group (*P* < 0.05). After treatment, DQYT, STW-M, and STW-H could attenuate the pregnancy loss (*P* < 0.05). Moreover, no significant difference was noted between the model and STW-L groups (Table 1).

After delivery, the average litter size was counted, the offspring were measured and weighed every 3 days, and the length and weight curves were recorded. The results revealed that the number of offspring per mouse in the model group decreased relative to that in the control group (*P* < 0.05), while the number of offspring per mouse in the DQYT, STW-H, STW-M, and STW-L groups increased relative to that in the model group (*P* < 0.05). In addition, the number of offspring per mouse in the STW-H and STW-M groups increased relative to that in the STW-L group (*P* < 0.05) (Table 2). Thus, as seen from the growth curve of the offspring, the length and weight of the offspring in the model group decreased relative to that in the control group, especially on 15–21 days, and the length and weight of the offspring in the DQYT, STW-H, and STW-M groups increased relative to those in the model group (*P* < 0.05), indicating good growth and development in the former (Figure 2).

### 3.2. Effect of STW on the Levels of P and CG in RSA Mice

The serum P and CG levels were measured by the ELISA on the 6^th^ day of pregnancy. The results revealed no significant difference in the serum P and CG levels between the groups (*P* > 0.05) (Table 3).

### 3.3. STW Improves the Morphology of Trophoblast Cells in the Blastocyst of RSA Mice

In the control group, trophoblast cells of the pregnant mice had regular morphology, neat arrangement, clear structure, abundant cytoplasm, acidic change, large nucleoli, and abundant blood vessels in the interstitium. In the model group, trophoblasts became irregular in shape, scattered in arrangement, and unclear in structure, indicating scattered basophilic changes in the cytoplasm, nuclear consolidation, and fragmentation, as well as a small amount of nuclear disappearance with reduced numbers of interstitial blood vessels. The morphology and structure of trophoblasts were improved after the intervention of dydrogesterone or STW. The improvement effect of dydrogesterone and the moderate- and high-dose STW was more evident, with more regular cell morphology, clearer structure, and neater arrangement, with a few cells showing consolidated and fragmented nuclei and relatively more abundant interstitial blood vessels (Figure 3).

### 3.4. STW Promotes Lactate Production in the Blastocysts of RSA Mice

The blastocyst tissues of the pregnant mice in each group were collected on the 6^th^ day for the determination of lactate content. The results indicated that the lactate content in the blastocyst tissues of the model group decreased when compared with that in the control group (*P* < 0.05). The lactate content in the blastocyst tissues of the DQYT, STW-H, and STW-M groups increased when compared with that in the model group (*P* < 0.05. The lactate content in the blastocyst tissues of the STW-H and STW-M groups increased when compared with that in the STW-L group (*P* < 0.05), albeit there was no statistically significant difference between the STW-H and STW-M groups in these terms (*P* > 0.05) (Figure 4).

### 3.5. Effect of STW on ATP Production in the Blastocysts of RSA Mice

The blastocyst tissues of the pregnant mice in each group were collected on the 6^th^ day for the determination of the ATP content. The results revealed that the ATP content in the blastocyst tissues of the model group increased when compared with that in the control group (*P* < 0.05). The lactate content in the blastocyst tissues of the STW-H, STW-M, and STW-L groups increased when compared with that in the model group (*P* < 0.05). The ATP content of the blastocyst tissues in the STW-H, STW-M, and STW-L groups decreased when compared with that in the model group (*P* < 0.05); however, there was no significant difference in the DQYT group (*P* > 0.05). In addition, the ATP content in the blastocyst tissues of the STW-H and STW-M groups decreased when compared with that in the STW-L group (*P* < 0.05), albeit there was no significant difference between the STW-H and STW-M groups in these terms (*P* > 0.05) (Figure 5).

### 3.6. Regulatory Effect of STW on the LDH, HK, and PK Enzyme Activities in the Blastocyst of RSA Mice

In order to explore the regulatory effect of STW on glycolysis, the effects of STW on the activities of key enzymes HK, PK, and LDH in glycolysis were detected by the colorimetric assay. A prominent decrease was noted in the HK enzyme activity in the model group when compared with that in the control group (*P* < 0.05). However, after dydrogesterone and high-dose STW treatment, this trend was reversed (*P* < 0.05) (Figure 6(a)). The PK enzyme activity in the model group increased when compared with that in the control group (*P* < 0.05). However, there was a decrease in the PK enzyme activity in the DQYT, STW-H, STW-M, and STW-L groups compared with that in the model group (*P* < 0.05). Among these, high-dose STW showed the best improvement effect (*P* < 0.05) (Figure 6(b)). The LDH enzyme activity was decreased in the model group compared with that in the control group (*P* < 0.05), while dydrogesterone and STW treatment showed improvement in the LDH enzyme activity (*P* < 0.05). The expression of the LDH enzyme activity in the STW high-dose group was similar to that in the STW moderate-dose group (*P* > 0.05) (Figure 6(c)).

### 3.7. Regulatory Effect of STW on the Expression Levels of HK2, PKM2, And LDHA in Blastocyst of RSA Mice

TRPO2 is a specific marker of trophoblasts; therefore, the glycolysis levels of different groups of trophoblasts were determined by immunofluorescence double staining using a mixture of target and TROP2 antibodies. Nuclear DAPI staining was blue, HK2, PKM2, and LDHA-positive proteins were green, and TROP2-positive protein was red. The protein expression level of HK2 was notably reduced in the model group than in the control group (*P* < 0.05); however, all treatment groups could facilitate its expression (*P* < 0.05). Moreover, the protein expression level of HK2 in the STW-M group was increased compared with that in the STW-L and STW-H groups (*P* < 0.05) (Figure 7(a) and 7(d)). Immunofluorescence results revealed a significant decrease in the PKM2 protein level in the model group compared with that in the control group (*P* < 0.05); however, treatment with dydrogesterone, STW-H, and STW-M could promote it (*P* < 0.05), albeit there was no statistically significant difference between the three groups (*P* > 0.05) (Figure 7(b) and 7(e)). The LDHA protein level was much lower in the model group than that in the control group (*P* < 0.05), and it could be inhibited by DQYT, STW-H, and STW-M treatment (*P* < 0.05). However, there was no significant difference in the LDHA protein expression between the STW-H and STW-M groups (*P* > 0.05) (Figure 7(c) and 7(f)).

### 3.8. Regulatory Effect of STW on the Expression Levels of GLUT1, MCT4, and GPR81 in Blastocyst of RSA Mice

Next, we examined GLUTI, which is responsible for glucose uptake. As shown in Figure 8(a), GLUT1 immunoreactivity was evident in trophoblasts, and the GLUT1 levels were decreased in the model group when compared with those in the control group (*P* < 0.05); however, it could be inhibited by DQYT, STW-H, and STW-M treatments (*P* < 0.05). Furthermore, the expression pattern of GLUT1 mRNA was consistent with that of the GLUT1 protein (*P* < 0.05) (Figure 9(a)). Subsequently, we examined MCT4, which is responsible for lactate transport, and immunofluorescence revealed that the MCT4 protein level was lower in the model group than that in the control group (*P* < 0.05). DQYT, STW-H, STW-M, and STW-L treatments elevated the MCT4 level (*P* < 0.05) (Figure 8(b) and 8(d)). On the other hand, the quantification of MCT4 mRNA implied a similar trend for the MCT4 protein level (Figure 9(b)). Finally, we examined the mRNA expression level of the lactate receptor GPR81, and it was found that compared with the control group, the expression of GPR81 mRNA in the model group was decreased (*P* < 0.05), which could be rescued after DQYT, STW-H, and STW-M treatments (*P* < 0.05) (Figure 9(c)).

## 4. Discussion

In the early pregnancy stage, embryo implantation is considered to be one of the most critical steps that have a decisive impact on successful pregnancy [11]. Implantation is divided into three stages: attachment, adhesion, and penetration. In the attachment stage, the connection of the trophoblast to the luminal epithelium is insufficiently tight. Subsequently, intimate adherence of the trophectoderm to the luminal epithelium occurs on day 4 at midnight [9]. After adhesion, the embryo invades the stroma via the luminal epithelium from the evening of day 5 to the morning of day 6, thus establishing a relationship with the maternal vasculature [12]. Therefore, in this experiment, the 6^th^ day after pregnancy was selected for the study. The decidua can limit the extent of invasion during this process, but it is predominantly controlled by trophoblasts [13]. In the early stages of normal pregnancy, invasive extravillous trophoblasts (EVTs) migrate into the maternal uterus and modify the blood vessels [14]. Failures in this process have been noted in RSA [15]. It is crucial to select an appropriate RSA animal model for specific mechanism studies. In this research, the CBA/J^*∗*^DBA/2 mouse model was selected because it is a miscarriage model that belongs to peri-implantation abortion, and the abortion rate is relatively constant [16].

STW is a classic herbal formula for the treatment of RSA. In the past 10 years, there have been thousands of clinical reports establishing the effectiveness of STW in RSA [2]. This study intended to reveal the possible mechanism of STW in the treatment of RSA. P is a hormone necessary for the establishment and maintenance of pregnancy in humans [17, 18]. In patients with three or more consecutive miscarriages immediately before the current pregnancy, empiric progestogen administration may be of some potential benefit in reducing the miscarriage rate [18–20]. Therefore, we selected dydrogesterone as the control medicine in this experiment. Chinese medicine emphasizes the idea of “prevention before disease onset [21].” The treatment of RSA focuses on “compensating weakness in advance” before the pregnancy, especially the kidneys and spleen, and protecting the fetus as soon as possible after the pregnancy occurs [22, 23]. This concept is similar to that of preventive medicine in Western medicine [24]. Because it takes 85 days for the follicles to grow and develop from preantral follicles to mature follicles, which spans three menstrual cycles, many doctors recommend that the treatment of patients with RSA be started at least 3 months before pregnancy and that targeted preventive treatment be administered before pregnancy [25]. In this study, the female mice in the RSA model group were treated with the medicine from 14 days before gestation to 6 and 14 days after gestation to achieve the effect of prepregnancy prevention and postpregnancy tocolysis.

In our research, the embryo loss rates were 6.12% in the control group and 33.33% in the model group. Compared with the control group, the embryo loss rate was significantly higher in the model group. However, after treatment with either dydrogesterone or high, medium, and low doses of STW, the embryo loss rate was significantly decreased. This result agrees with that of other studies. Zeng's research [2] found that when compared with the model group, the embryo loss rate was significantly lower in the STW high-dose group and medium-dose group. This study predicted the potential targets of STW in humans using proteomic tools and confirmed that STW can regulate the expression of various proteins in the decidua of RSA mice, such as desmin involved in the invasion and transformation of trophoblasts and muscular spiral arteries. Another study showed that STW can improve the pregnancy rate by improving uterine receptivity and providing a good environment for embryo implantation [26]. Animal experimental studies often use the pregnancy rate and the embryo loss rate as the pregnancy outcomes [2], whereas clinical studies follow up on all infants for malformations and developmental abnormalities for 6 months after delivery [27]. Therefore, unlike other experiments, this study examined the effect of STW on the number and growth of offspring. The results showed that STW could increase the number of offspring and promote their growth and development, suggesting that it has a significant tocolytic effect.

It is well known that P plays a vital role in maintaining early pregnancy in humans. The hormone not only maintains adequate decidualization of the endometrium during pregnancy but also acts as a major immune determinant and controls uterine contractility and cervical function [17, 28]. Moreover, studies have shown that human chorionic gonadotropin (hCG) promotes placental cell differentiation and angiogenesis and induces the production of specific matrix metalloproteinases that promote the invasion of trophoblasts into the endometrium [29]. An in vitro cell experiment showed that serum containing STW can dose dependently enhance *β*-hCG secretion [30]. However, in our study, significant differences were not observed in the levels of P and CG between the RSA model group and the control group. Furthermore, the treatment with dydrogesterone and STW did not affect the expression levels of these two hormones. Hence, the mechanism of STW increasing the pregnancy rate in the RSA model mice may be independent of P and CG. However, whether STW has a regulatory effect on the receptors of two hormones remains to be explored.

Proper trophoblast invasion and proliferation are critical for embryo implantation and placental development, which facilitate the establishment of a proper maternal-fetal relationship. The invasive/proliferative properties of extravillous trophoblasts are known to be abnormally reduced under pathological conditions [31], and the precise execution of various functions of trophoblasts directly affects embryo survival [32]. Studies have shown that serum containing STW can enhance the proliferative activity, migration, and invasion ability of trophoblast cells and reduce the apoptosis of trophoblast cells [30]. In this study, HE staining results showed that the morphology of the trophoblasts in the RSA model mice was abnormal. Moreover, the abnormal cell structure during pregnancy may affect the invasion and migration ability of trophoblasts, thus resulting in miscarriage [33]. Dydrogesterone and STW treatment could improve the morphology of trophoblast cells, thereby protecting the embryo.

Trophoblasts participate in embryo implantation by sensing the alterations in the uterine microenvironment and regulating maternal-fetal immune tolerance and invasive capacity. The uterine environment is hypoxic during the peri-implantation period of pregnancy, which affects the utilization of specific metabolic pathways that favor the organism's growth and survival [34]. Trophoblasts, like cancer cells, use aerobic glycolysis as the major metabolic pathway even in the presence of oxygen [35]. A major metabolite of aerobic glycolysis is lactate, which creates a specific microenvironment characterized by high lactate levels at implantation and reduced pH around the blastocyst [5]. Moreover, lactate is a key mediator of the maternal-fetal dialogue that supports implantation [6]. This study revealed that the embryonic lactate content of the RSA model mice was reduced. Hence, the microenvironment of embryo implantation with high lactate and low pH was destroyed, which suggests that the pathogenesis of RSA may be related to the insufficient level of aerobic glycolysis. However, a recent study has contradicted our findings and reported an enhancement of the lactate microenvironment in patients with RSA compared with normal pregnancies. Presumably, the decidual microenvironment in patients with RSA is more prone to hypoxia, and thus, the decidua increases lactate production via anaerobic glycolysis [36]. Interestingly, another study has supported our findings. The contents of lactate and pyruvate in the villi of patients with RSA were lower than those of patients who terminated the pregnancy for nonmedical reasons, implying that changes in the glycolytic metabolism of villi are related to the occurrence of RSA [31]. Furthermore, the ATP contents of the embryos were measured in the present study, and the ATP content of the RSA model mice was significantly higher than that of the control group. However, mitochondrial activity is not essential for early embryo growth and proliferation before postfertilization day 8.5 [37]; therefore, the elevated ATP content in the RSA model mice may not be a favorable phenomenon. The Warburg effect is less efficient in generating ATP compared with oxidative phosphorylation, but it effectively meets the need for the production of macromolecules, such as nucleic acids, to promote cell proliferation [38]. After treatment with dydrogesterone and different doses of STW, the levels of lactate and ATP in the RSA model mice were improved to varying degrees, thereby correcting the decreased levels of glycolysis and the production of macromolecules in the RSA model mice. Among them, moderate-dose and high-dose STW had the best effect, and there was no significant difference between the two groups. We intend to further explore the abnormal aerobic glycolytic process in RSA and the regulatory effect of STW on aerobic glycolysis.

Aerobic glycolysis comprises three irreversible steps that are regulated by HK or glucokinase (GCK), phosphofructokinase (PFK), and PK. In this study, the activities of the key enzymes involved in aerobic glycolysis were measured in mouse embryonic trophoblasts, including HK, PK, and LDH. Simultaneously, the protein expression levels of enzymes, including HK2, PKM2, and LDHA, were determined. The results showed that the activities of HK and LDH decreased and that the protein expression levels of HK2 and LDHA decreased in the RSA model mice. HK is the first rate-limiting enzyme in the glycolytic pathway, and HK2 is highly expressed in embryos cultured under hypoxic conditions to support aerobic glycolysis [39]. LDHA catalyzes the conversion of pyruvate to lactate and maintains elevated NAD^+^ levels to support glycolysis [38]. Furthermore, its expression is positively correlated with the Warburg effect. PK is the ultimate rate-limiting enzyme in the aerobic glycolysis pathway, and PKM2 is predominantly expressed in embryonic tissues and proliferating cells [40]. This study found increased PK activity in the trophoblasts of the RSA model mice; however, the expression levels of PKM2 protein were decreased. Studies have reported that the expression of PKM2 is closely related to tumor cell proliferation and differentiation [41, 42]. Therefore, PKM2 is speculated to be involved in the embryo implantation process. The less active dimeric form of PKM2 promotes aerobic glycolysis, converts pyruvate to lactate for energy production, and permits the redistribution of glycolytic intermediates to support macromolecule biosynthesis and cell proliferation [43]. Collectively, the findings demonstrate that the pathogenesis of RSA miscarriage may be related to the abnormal activity and expression levels of key enzymes in aerobic glycolysis, thereby inhibiting aerobic glycolysis and affecting the embryo implantation process. After dydrogesterone or STW intervention, the activities of HK and LDH enzymes as well as the expressions of HK2 and LDHA proteins increased. The elevated expression of PKM2, despite the expression of the less active isoform, led to an overall increase in the glycolytic flux, thereby resulting in higher flux through PKM2. The findings from this study show that STW can promote aerobic glycolysis by regulating the activities and expression levels of key enzymes in aerobic glycolysis, thus improving the microenvironment and promoting embryo implantation.

Glucose is the major energy substrate used by trophoblasts, and GLUT1 is the rate-limiting enzyme in glucose metabolism responsible for basal glucose uptake by these cells [44, 45]. The transition from aerobic oxidative metabolism to hypoxic glycolysis is one of the hallmarks of cancer cells, and the overexpression of GLUT1 promotes the adaptive upregulation of tumor glycolysis [39]. Owing to similarities in the characteristics of trophoblasts and cancer cells, the expression level of GLUT1 in trophoblasts is speculated to represent the level of glycolysis to some extent. In the present study, the expression of GLUT1 in trophoblast cells and its potential role in the pathogenesis of RSA were investigated. The data demonstrate that mRNA and protein levels of GLUT1 are significantly reduced in the trophoblasts of RSA mice, which suggests that Warburg-like glycolysis is impaired in RSA. Evidence also alludes that the inhibition of the Warburg effect reduces cell growth, thereby inducing apoptosis of placental trophoblastic cells and ultimately leading to early miscarriage. As a glucose uptake pump, downregulation of GLUT1 results in decreased glucose utilization, an outcome that can be rescued by dydrogesterone or STW treatment. When cells undergo glycolysis, intracellular lactate needs to be transported to the outside of the cell to avoid negative feedback inhibition of glycolytic flux due to intracellular accumulation [46]. The function of lactate depends on specific receptors, and the major ones are monocarboxylate transporters (MCTs) and *G*protein-coupled receptors (GPRs). MCT4 is a low-affinity transporter of lactate and is chiefly expressed in highly glycolytic cells [47]. GPR81 acts as a lactate sensor that regulates the expression of lactate metabolism and transports genes according to the lactate concentration in the immediate environment [48]. The present findings assert that the expressions of MCT4 and GPR81 are decreased in the trophoblasts of the RSA mice and that STW can upregulate the expression levels of MCT4 and GPR81 in trophoblasts. MCT4 is responsible for exporting lactate out of the cell in response to high glycolytic flux and is upregulated in response to hypoxia, whereas GPR81 acts concertedly with lactate to facilitate implantation [47, 48].

Furthermore, a comprehensive analysis of the experimental results revealed that STW-M, which is equivalent to twice the dose commonly used in clinical settings, was more effective than STW-L, STW-H, and DQYT in increasing the level of aerobic glycolysis in trophoblasts. This result signifies that moderate doses of STW are suitable for the treatment of RSA and that they provide a certain value for guiding clinical medication.

## 5. Conclusions

The present findings revealed that insufficient aerobic glycolysis in the trophoblast cells in the RSA mouse model could result in an abnormal microenvironment, leading to embryo implantation failure. STW can improve the embryo implantation microenvironment by promoting high levels of aerobic glycolysis, thereby promoting embryo implantation (Figure 10). Cumulatively, these data contribute to our understanding of the important role of aerobic glycolysis in supporting and promoting implantation, which will be of great value in improving and establishing implantation success.

## Figures and Tables

**Figure 1:** Effects of STW on the mouse uterus and embryo morphology: (a) control group; (b) model group; (c) DQYT group; (d) STW-L group; (e) STW-M group; (f) STW-H group. Red arrows indicate lost embryos.

**Figure 2:** Effects of STW on the growth and development of offspring mice: (a) length curve of offspring of pregnant mice in each group; (b) body weight curve of offspring of pregnant mice in each group. Compared with the control group, ^*∗*^*P* < 0.05; compared with the model group, ^#^*P* < 0.05; compared with the DQYT group, ^△^*P* < 0.05.

**Figure 3:** Effects of STW on the morphology of trophoblasts in mouse embryos: (a) control group; (b) model group; (c) DQYT group; (d) STW-L group; (e) STW-M group; (f) STW-H group. The fetus with the uterus (5×) and the local trophoblast (63×).

**Figure 4:** Effects of STW on lactate content in blastocyst tissue of pregnant mice (*n* = 5). Compared with the control group, ^*∗*^*P* < 0.05; compared with the model group, ^#^*P* < 0.05 compared with the DQYT group, ^△^*P* < 0.05.

**Figure 5:** Effects of STW on ATP content in blastocyst tissue of pregnant mice (*n* = 3). Compared with the control group, ^*∗*^*P* < 0.05; compared with the model group, ^#^*P* < 0.05; compared with the DQYT group, △*P* < 0.05.

**Figure 6:** Effects of STW on the activities of HK, PK, and LDH enzymes in blastocyst tissue of pregnant mice (*n* = 4): (a) HK enzyme activity in blastocyst tissue of pregnant mice in each group; (b) PK enzyme activity in blastocyst tissue of pregnant mice in each group; (c) LDH enzyme activity in blastocyst tissue of pregnant mice in each group. Compared with the control group, ^*∗*^*P* < 0.05; compared with the model group, ^#^*P* < 0.05; compared with the DQYT group, ^△^*P* < 0.05.

**Figure 7:** Effects of STW on the expression levels of HK2, PKM2, and LDHA proteins in mouse trophoblasts (40×): (a) HK2 immunohistochemistry staining in trophoblasts; (b) PKM2 immunohistochemistry staining in trophoblasts; (c) LDHA immunohistochemistry staining in trophoblasts; (d–f) HK2, PKM2, and LDHA protein levels in trophoblasts. Compared with the control group, ^*∗*^*P* < 0.05; compared with the model group, ^#^*P* < 0.05; compared with the DQYT group, ^△^*P* < 0.05.

**Figure 8:** Effects of STW on the expression levels of GLUT1 and MCT4 proteins in mouse trophoblasts (40×): (a) GLUT1 immunohistochemistry staining in trophoblasts; (b) MCT4 immunohistochemistry staining in trophoblasts; (c–d) GLUT1 and MCT4 protein levels in trophoblasts. Compared with the control group, ^*∗*^*P* < 0.05; compared with the model group, ^#^*P* < 0.05; compared with the DQYT group, ^△^*P* < 0.05.

**Figure 9:** Effects of STW on the expression levels of GLUT1, MCT4, and GPR81 mRNA in mouse blastocyst tissue: (a) expression levels of GLUT1 mRNA in blastocyst tissues of pregnant mice in each group; (b) expression levels of MCT4 mRNA in blastocyst tissues of pregnant mice in each group; (c) expression levels of GPR81 mRNA in blastocyst tissues of pregnant mice in each group. Compared with the control group, ^*∗*^*P* < 0.05; compared with the model group, ^#^^*∗*^*P* < 0.05; compared with the DQYT group, ^△^^*∗*^*P* < 0.05.

**Figure 10:** The summary of this study. STW promotes the level of aerobic glycolysis in trophoblast cells and improves the microenvironment of embryo implantation in RSA mice, thereby promoting embryo implantation.

**Table 1:** Effects of STW on pregnancy outcomes on embryo day 14.

Group	Pregnant number	Total number of embryos	Number of viable embryos	Number of lost embryos	Embryo loss rate (％)
Control group	6	49	46	3	6.12
Model group	6	48	32	16	33.33^*∗*^
DQYT group	6	49	43	6	12.24^#^
STW-L group	6	50	37	13	26^*∗*^
STW-M group	6	49	42	7	14.29^*∗*^
STW-H group	6	48	43	5	10.42^#^

Compared with the control group, ^*∗*^*P* < 0.05; compared with the model group, ^#^*P* < 0.05; compared with the DQYT group, ^△^*P* < 0.05.

**Table 2:** Effects of STW on the number of offspring of pregnant mice.

Group	Pregnant number	Average number of offspring
Control group	6	7.67 ± 0.33
Model group	6	2.67 ± 0.56^*∗*^
DQYT group	6	7.67 ± 0.49^#^
STW-L group	6	4.67 ± 0.42^*∗*^^#△^
STW-M group	6	6.17 ± 0.48^#^
STW-H group	6	7.33 ± 0.49^#^

Compared with the control group, ^*∗*^*P* < 0.05; compared with the model group, ^#^*P* < 0.05; compared with the DQYT group, ^△^*P* < 0.05.

**Table 3:** Effects of STW on serum P and CG in pregnant mice.

Group	P (ng/mL)	CG (IU/L)
Control group	0.99 ± 0.05	4.41 ± 0.05
Model group	1.10 ± 0.03	4.28 ± 0.12
DQYT group	1.11 ± 0.03	4.19 ± 0.09
STW-L group	1.05 ± 0.03	4.15 ± 0.05
STW-M group	1.07 ± 0.03	4.22 ± 0.10
STW-H group	1.10 ± 0.03	4.13 ± 0.09

## Data Availability

The datasets used and/or analyzed during the current study are available from the corresponding author upon reasonable request.
